The article "Study on Risk Factors and Nutritional Status of Postoperative Infection in Patients Undergoing Abdominal Surgery" was retracted in 2023. Reasons: signs of a paper mill; suspected computer-generated content; unreliable results or conclusions; lack of ethics approval or compliance.

# Study on Risk Factors and Nutritional Status of Postoperative Infection in Patients Undergoing Abdominal Surgery

**DOI:** 10.1155/2022/8063851

**Published:** 2022-07-19

**Authors:** Zhejin Wang, Chen Li, Qi Quan, Ying Zhang

**Affiliations:** ^1^Department of Hepatobiliary Surgery, Wenzhou Central Hospital, The Second Affiliated Hospital of Shanghai University, Wenzhou 325000, China; ^2^Department of Clinical Laboratory, Wenzhou Hospital of Integrated Traditional Chinese and Western Medicine, Integrated Traditional Chinese and Western Medicine Hospital Affiliated to Shanghai University, Wenzhou 325000, China

## Abstract

In order to evaluate the risk factors of postoperative infection in patients undergoing abdominal surgery and the correlation with nutritional status, 143 patients admitted to our hospital for abdominal surgery from September 2020 to September 2021 are selected and analyzed. By collecting the clinical results and related pathological data of all patients, all patients are divided into the postoperative infection group (48 cases) and the noninfection group (95 cases) according to whether postoperative infection occurred. Firstly, the clinical data of the two groups are analyzed by univariate analysis. Secondly, the risk factors of postoperative infection in patients undergoing abdominal surgery are analyzed by binary logistic regression. Thirdly, the nutrition-related indexes are compared, and the correlation between postoperative infection and serum nutritional indexes is analyzed by the Spearman correlation coefficient. The results demonstrate that patients undergoing abdominal surgery have a certain risk of infection after surgery, and combination with underlying diseases is a risk factor for postoperative infection. In addition, poor preoperative nutritional status is also closely related to postoperative infection. It is suggested that serum PA and RBP indicators have certain predictive effects on postoperative infection.

## 1. Introduction

Postoperative infection is one of the common complications of abdominal surgery. If a patient has adverse complications such as infection after abdominal surgery, it will not only affect the clinical rehabilitation utility of the patient but also reduce the surgical effect on the patient. Due to the increase in adverse reactions of patients, the hospitalization time for patients was significantly prolonged. This further increases the clinical hospitalization expenses of patients, increases the economic pressure on patients and their families in disease treatment, and brings two-way physical and mental pain to patients [1, 2]. Clinical research data show that the proportion of hospital infections in surgical inpatients is high. For clinical abdominal surgery patients, poor resistance, large subcutaneous fat thickness, and postoperative subcutaneous hemorrhage make them prone to fat liquefaction and other adverse symptoms. This is an important mechanism of postoperative infection, which seriously affects the prognosis of patients. Without timely intervention, the deterioration of the patient's infection symptoms may further lead to systemic infection. In serious cases, patients may face risks such as multiple organ dysfunction and are very likely to have adverse events [3, 4].

The consequence of abdominal infection after the operation is related to the patient's condition, treatment opportunity, and other factors. The main manifestations were peritonitis and abdominal abscess [5]. Moreover, more than 90% of primary peritonitis is caused by a single bacterium. The most common pathogen was Gram-negative bacilli, followed by *Streptococcus pneumoniae*, accounting for 15% [6]. Secondary peritonitis is usually caused by perforation or necrosis of hollow organs or bacterial dissemination in the abdominal cavity. The upper digestive tract is dominated by Enterobacteriaceae bacteria, and the lower digestive tract is perforated or broken [7]. The bacterial pollution is relatively serious, and mixed infection including anaerobic bacteria is common. Most of the pathogens of the third type of peritonitis are drug-resistant bacteria, including *Enterococcus*, *Candida albicans*, *Staphylococcus epidermidis*, *Pseudomonas aeruginosa*, *Acinetobacter baumannii*, and fungi [8, 9]. The abdominal abscesses in the lower diaphragm and upper abdomen are mainly Enterobacteriaceae. The lower abdominal and pelvic abscesses were mainly anaerobic fragile Bacteroides and aerobic Enterobacteriaceae, as well as other bacteroides and clostridium.

This paper is organized as follows.  Section 2 discusses the related work, followed by our proposed methods and statistical processing in Section 3. In section 4, the results and analysis are proposed. Finally, in Section 5, some concluding remarks are made.

## 2. Related Work

Previous studies have shown that patients undergoing abdominal surgery have a high proportion of postoperative infection [10]. In recent years, with the continuous progress of medical technology, abdominal surgery gradually tends to be minimally invasive, helping many clinical patients to receive relevant diagnosis and treatment as soon as possible [11]. It is important to note that abdominal surgery in patients with postoperative complications risk remains high, and postoperative infection prevention and control is particularly important. The popularity of abdominal surgical minimally invasive surgery allows a lot of abdominal surgery patients to early and timely treatment, but the control of postoperative patients with all kinds of complications and the emphasis is still an inadequate investment. The most prominent one is the control of postoperative pulmonary infection. Therefore, it is necessary to analyze the clinical characteristics and related risk factors of patients with postoperative infection after abdominal surgery for the prevention and treatment of postoperative complications [12].

The results of this study were compared and analyzed on the related factors of postoperative infection in patients with abdominal surgery and showed that age ≥60 years, surgical incision length ≥10 cm, surgical duration ≥2 h, length of hospital stay ≥10 d, and combined underlying diseases were the risk factors for postoperative infection in patients with abdominal surgery. Based on the analysis of the reasons for the above research results, with the increase of age, the body function of patients is increasingly degraded, and the immune function is reduced. After abdominal surgery, the body resistance is reduced, which is prone to infection and other complications [13]. With basic diseases such as diabetes mellitus patients, as a result of their disease influence white blood cell function is impaired, the immunity worsens, further reducing anti-infection ability, and patients with hypertension are affected by abnormal blood pressure index, which affects local blood circulation at the surgical site after operation and delays wound healing [14, 15]. Some studies showed that the long operation time inevitably brings about long incision length. In addition, the more serious the patient's tissue damage is, the longer the operation time will increase the number and exposure of wound bacteria. The long operation time may lead to the decline of patients' immunity and endogenous infection. Moreover, it will lead to a relatively long postoperative recovery time and increase the risk of postoperative infection. The results of this study are basically consistent with those of previous studies [16]. According to the risk factors of surgical incision infection, preventive intervention measures should be taken. Antibiotics were used routinely after the operation, and the dressing change frequency was increased. For the elderly and infirm patients with basic diseases, nutrition should be strengthened to improve their own immunity. In addition, try to adjust the operation to the most appropriate conditions and select the most appropriate operation method to reduce the operation time and incision length. This will help to shorten incision exposure time and reduce the chance of infection [17].

In addition, this study conducted an in-depth analysis of postoperative infection of patients with abdominal surgery and their nutritional status, indicating that the concentration of serum nutritional indexes PA and RBP is closely related to postoperative infection. In recent years, the concept of accelerated postoperative recovery has been widely valued and applied in surgical nursing management. Clinicians are paying more and more attention to the perioperative management of patients and gradually realize that nutritional status has a huge impact on postoperative rehabilitation [18]. After postoperative infection, the proportion of patients with malnutrition increased greatly due to a long bedtime and decreased gastrointestinal digestive and absorption functions, nutritional intake disorders, trauma and surgical stress, wound healing needing extra energy, and other reasons [19]. Recent research results suggest that, before the condition permits, the intake of nutrients and energy through the digestive tract is still the best way. It has positive effects to pay attention to and improve the nutritional status of patients, enhancing the secretion level of hormones related to the intestinal and digestive organs and maintaining the balance of intestinal flora and immune function [20].

To sum up, in the clinical work of patients undergoing abdominal surgery, we need to focus on their age and body immune function, cooperate with basic diseases, incision length, operation time, hospital stay, strictly control the independent risk factors affecting infection, and take measures to do a good job in anti-infection from many aspects, so as to effectively reduce the risk of postoperative infection. In addition, there are still nutritional risks in patients undergoing abdominal surgery. Strengthening nutritional risk screening and providing targeted nutritional support to patients can help improve patients' nutritional reserve, avoid nutritional risk deterioration, reduce the incidence and severity of postoperative infection, and accelerate postoperative recovery.

## 3. Our Proposed Methods and Statistical Processing

A total of 143 patients, including 81 males and 62 females, aged 26–72 years, with an average of (49.26 ± 7.68) years, were selected from September 2020 to September 2021. Among them, 74 patients received gastrointestinal surgery, and 58 patients received hepatobiliary, pancreatic and splenic-related surgery. A total of 17 patients received other types of operations.

Inclusion criteria are as follows: (1) patients were indicated by clinicopathology and related diagnosis; (2) complete clinicopathological data of patients; (3) patients with high clinical compliance can cooperate with this study to complete relevant investigation until the end of the study; (4) patients have clear consciousness and no mental diseases such as cognitive impairment.

Exclusion criteria are as follows: (1) patients with malignant tumor-related diseases; (2) before admission to our hospital, she had received relevant out-of-hospital operations; (3) patients with mental illness or signs of consciousness disorder; (4) patients who dropped out of the study for various reasons.

### 3.1. Investigation Methods of Patient-Related Information

All patients admitted to hospital after collecting their name, sex, age, body mass index (BMI), and other basic information, hospital during the period of treatment to collect the patients' surgical site, operation time, intraoperative incision at base type, length of hospital stay, the body condition, such as data, and analysis of the above indicators whether postoperative infection in patients with abdominal surgery.

### 3.2. Postoperative Infection Detection Method

After surgery, all patients' deep wound secretions were collected by sterilized cotton swabs before medication, placed in sterile test tubes, and sent to a pathogen microbial laboratory. All samples were inoculated in a blood agar plate and cultured in a 35°C incubator for 24–72 h. ATB automatic microbial analyzer and supporting reagents were used. Meili YI API identification strip was used for microbial identification, Meili Yi ATB drug-sensitive strip was used for drug sensitivity test, and the results were interpreted by naked eyes. According to the “National Standard of Clinical Inspection Operation,” ATCC25922 *Escherichia coli*, ATCC27853 *Pseudomonas aeruginosa*, and ATCC25923 *Staphylococcus aureus* were used for quality control.

### 3.3. Methods for Diagnosis of Postoperative Infection

All patients with postoperative infection were diagnosed according to the Hospital Infection Diagnostic Criteria issued by the Ministry of Health [21]. Patients with postoperative infection were included in the postoperative infection group (*n* = 48), and patients without infection were included in the noninfection group (*n* = 95). There were no statistically significant differences between the two groups in operating room preparation, instrument disinfection, preoperative preparation, perioperative nursing, and anesthesia mode (all *P* > 0.05), indicating comparability.

8 mL of fasting peripheral venous blood was collected from both groups. Nutritional biochemical parameters including prealbumin (PA), albumin (ALB), hemoglobin (Hb), and retinol-binding (RETINol binding) were analyzed by an AU5800 automatic biochemical analyzer (Beckman Kuhl, USA) Protein, RBP, and other serum concentrations were used to evaluate the nutritional status of patients after surgery.

### 3.4. Observation Indicators

The observation indicators are as follows: (1) univariate analysis of clinicopathological data; (2) binary logistic regression analysis of risk factors for postoperative infection in patients undergoing abdominal surgery; (3) postoperative nutritional indexes were compared; (4) the correlation between postoperative serum nutritional indexes and infection was analyzed.

### 3.5. Statistical Processing

SPSS 26.0 analysis and processing software was used to integrate all the data in this study, measurement data was expressed as ($\bar{x}\pm s$), intergroup comparison was performed by *t*-test, the rate of counting data was expressed by *χ*^2^ test, and the risk factors of postoperative infection in patients with abdominal surgery were studied by binary logistic regression analysis. Spearman correlation coefficient was used to analyze the correlation between patients' nutritional status and postoperative infection, and *P* < 0.05 indicated a statistically significant difference.

## 4. Analysis of Clinical Data and Results

### 4.1. Univariate Analysis of Clinicopathological Data

There are no significant statistical differences in clinical data, including gender, BMI, and incision type (all *P* > 0.05). As shown in Table 1, there are significant statistical differences in age, incision length, operation time, hospital stay, and basic diseases (all *P* < 0.05).

### 4.2. Binary Logistic Regression Analysis of Risk Factors for Postoperative Infection in Patients Undergoing Abdominal Surgery

Factors with *P* < 0.05 in single factors were taken as independent variables, postoperative infection in patients was included independent variables, and the variable assignment is shown in Table 2. Binary logistic regression analysis showed that the risk factors for postoperative infection in patients undergoing abdominal surgery included the following: age ≥60 years, surgical incision length ≥10 cm, operation time ≥2 h, hospital stay ≥10 d, and combination of basic diseases.

### 4.3. Nutritional Index Levels of Patients

Laboratory tests of serum nutritional indexes showed that PA and RBP in the postoperative infection group decreased significantly more than in the noninfection group (all *P* < 0.05). It can be observed from Table 3 that there was no significant difference in serum ALB and Hb concentrations (*P* > 0.05).

### 4.4. Analysis of the Correlation between Postoperative Serum Nutritional Indicators and Postoperative Infection

Spearman correlation coefficient analysis was carried out between *P* < 0.05 in serum nutritional indexes and the occurrence of postoperative infection. As shown in Table 4, serum PA and RBP were significantly negatively correlated with postoperative infection (*P* < 0.05).

## 5. Conclusions

In this study, the risk factors and nutritional status of postoperative infection in patients undergoing abdominal surgery are investigated. The clinical data of the two groups were analyzed by univariate analysis, and the risk factors of postoperative infection in patients undergoing abdominal surgery were analyzed by binary logistic regression. Furthermore, the nutrition-related indexes were compared, and the correlation between postoperative infection and serum nutritional indexes was analyzed by the Spearman correlation coefficient. From the experimental result, it demonstrates that the patients undergoing abdominal surgery will face a certain risk of infection after surgery. It is clearly evident that serum PA and RBP indicators have certain predictive effects on postoperative infection, and the targeted measures should be taken according to relevant risk factors to prevent postoperative infection. Therefore, emergency patients, elderly patients, and patients with long incisions improve the nursing risk level. For obese and overweight people, health education should be done well, and attention should be paid to body position management and skin care. Sweat stains should be cleared in time to avoid incision compression.

## Figures and Tables

**Table 1:** Univariate analysis of clinicopathological data.

Factors	Postoperative infection group (*n* = 48)	Uninfected group (*n* = 95)	*t*/*χ*^2^	*P*
Gender (*n*, %)			0.180	0.671
Male	26 (54.17)	55 (57.89)		
Female	22 (45.83)	40 (42.11)		

Age (*n*, %)			17.604	<0.001
≥60 years of age	35 (72.92)	34 (35.79)		
<60 years of age	13 (27.08)	61 (64.21)		

BMI (kg/m^2^)	23.12 ± 2.29	22.85 ± 2.14	0.696	0.488

Type of incision (*n*, %)			1.042	0.743
I	1 (2.08)	19 (20.00)		
II	22 (45.83)	37 (38.95)		
III	25 (52.09)	39 (41.05)		

Surgical incision length (*n*, %)			10.827	0.001
≥10 cm	15 (31.25)	9 (9.47)		
<10 cm	33 (68.75)	86 (90.53)		

The operation time (*n*, %)			21.020	<0.001
≥2 h	34 (70.83)	29 (30.53)		
<2 h	14 (29.17)	66 (69.47)		

The length of time (*n*, %)			26.223	<0.001
≥10 d	36 (75.00)	32 (33.68)		
<10 d	9 (18.75)	63 (66.32)		

Underlying medical conditions (*n*, %)			6.988	<0.001
Yes	25 (52.08)	28 (29.47)		
No	23 (47.92)	67 (70.53)		

**Table 2:** Variable assignment table.

Factors	The variable name	The assignment
Age (years)	*X*1	<60 years of age = 0, ≥60 years of age = 1
Surgical incision length (cm)	*X*2	<10 cm = 0, ≥10 cm = 1
The operation time (h)	*X*3	<2 h = 0, ≥2 h = 1
The length of time (d)	*X*4	<10 d = 0, ≥10 d = 1
Underlying diseases	*X*5	No = 0, yes = 1
Postoperative infection occurs	*Y*	No = 0, yes = 1

**Table 3:** Comparison of serum nutritional indexes ($\bar{x}\pm s$).

Group	PA (g/L)	ALB (g/L)	Hb (g/L)	RBP (g/L)
Postoperative infection group (*n* = 48)	132.18 ± 19.04	37.28 ± 3.72	126.03 ± 16.39	18.32 ± 3.73
Uninfected group (*n* = 95)	145.72 ± 20.27	36.33 ± 3.85	127.11 ± 17.32	21.04 ± 4.26
*t*	−3.848	1.409	−0.358	−3.761
*P*	<0.001	0.161	0.721	<0.001

**Table 4:** Correlation analysis between serum PA and RBP and postoperative infection in patients.

	Postoperative infection occurs	
	rs	*P*
PA (g/L)	−0.614	<0.001
RBP (g/L)	−0.589	<0.001

## Data Availability

The simulation experiment data used to support the findings of this study are available from the corresponding author upon request.

## References

[1] Meyer J., Roos E., Abbassi Z., Buchs N. C., Ris F., Toso C. (2020). Prophylactic negative-pressure wound therapy prevents surgical site infection in abdominal surgery: an updated systematic review and meta-analysis of randomized controlled trials and observational studies. *Clinical Infectious Diseases*.

[2] Vogelsang H., Lang A., Cevik B., Botteck N. M., Weber T. P., Niescery J. H. (2020). Incidence of infection in non‐tunnelled thoracic epidural catheters after major abdominal surgery. *Acta Anaesthesiologica Scandinavica*.

[3] Couture T., Gaudric J., Davaine J. M., JayetChicheJarrayaKoskas F. (2021). Results of cryopreserved arterial allograft replacement for thoracic and thoracoabdominal aortic infections. *Journal of Vascular Surgery*.

[4] Re A. M. D., Wright D., Toh J. (2021). Surgical wound infection prevention using topical negative pressure therapy on closed abdominal incisions-the “SWIPE IT” randomised clinical trial. *Journal of Hospital Infection*.

[5] Momin A. A., Barksdale E. M., Lone Z. (2020). Exploring perioperative complications of anterior lumber interbody fusion in patients with a history of prior abdominal surgery: a retrospective cohort study. *The Spine Journal*.

[6] Zhang L., Liu Y., Gao X. (2021). Immediate vs. gradual advancement to goal of enteral nutrition after elective abdominal surgery: a multicenter non-inferiority randomized trial. *Clinical Nutrition*.

[7] Simona S., Rosalba L., Alessio M. (2021). Procalcitonin and early postoperative infection after pediatric cardiopulmonary bypass surgery. *Journal of Cardiothoracic and Vascular Anesthesia*.

[8] Cals F. L. J., Toom H. F. E. V. D., Metselaar R. M., Linge A. V., Schroeff M. V. D., Pauw R. (2022). Postoperative surgical site infection in cholesteatoma surgery with and without mastoid obliteration, what can we learn?. *Journal of otology*.

[9] Lytvyn L., Quach K., Banfield L., Johnston B. C., Mertz D. (2016). Probiotics and synbiotics for the prevention of postoperative infections following abdominal surgery: a systematic review and meta-analysis of randomized controlled trials. *Journal of Hospital Infection*.

[10] Willinge G. J. A., Hietbrink F., Leenen L. P. H. (2021). Surgical airway procedures in emergency surgical patients: results of what has become a back-up procedure. *World Journal of Surgery*.

[11] Benoist H., Rodier S., Blanchardière A. D. L. (2019). Appropriate use of antifungals: impact of an antifungal stewardship program on the clinical outcome of candidaemia in a French University Hospital. *Infection*.

[12] McLean K. A., Mountain K. E., Shaw C. A., DrakeOtsKnightFairfieldSgròSkipworthWigmorePotterHarrison E. M. (2021). O8 Tracking wound infection with smartphone technology (twist): a randomised controlled trial in emergency surgery patients. *British Journal of Surgery*.

[13] Gan C., Wang Y., Tang Y., WangSunWangZhu F. (2021). Risk factors for surgical site infection in head and neck cancer. *Supportive Care in Cancer*.

[14] Bozzay J. D., Walker P. F., Schechtman D. W. (2021). Risk factors for abdominal surgical site infection after exploratory laparotomy among combat casualties. *Journal of the American College of Surgeons*.

[15] AlGamdi S. S., Alawi M. M., Bokhari R., BajunaidMukhtarBaeesa S. S. (2021). Risk factors for surgical site infection following spinal surgery in Saudi Arabia. *Medicine*.

[16] Nasser H., Ivanics T., Murali S. L., Stefanou A. (2020). Risk factors for surgical site infection after laparoscopic colectomy: an NSQIP database analysis. *Journal of Surgical Research*.

[17] McDougall R. A., Spector D. I., Hart R. C., DycusErb H. N. (2021). Timing of and risk factors for deep surgical site infection requiring implant removal following canine tibial plateau leveling osteotomy. *Veterinary Surgery*.

[18] Sakibul H., Khalafallah A. M., Adrian J. (2020). Nutritional status predicts hospital length of stay in meningioma patients. *Neurosurgery*.

[19] Ornaghi P. I., Afferi L., Antonelli A., CerrutoOdorizziGozzoMordasiniMatteiBaumeisterCorneliusTafuriMoschini M. (2021). The impact of preoperative nutritional status on post-surgical complication and mortality rates in patients undergoing radical cystectomy for bladder cancer: a systematic review of the literature. *World Journal of Urology*.

[20] Leung M. F., Wang J. (2022). Cardinality-constrained portfolio selection based on collaborative neurodynamic optimization. *Neural Networks*.

[21] Luo W. Y., Xu Z. M., Zhang Y. Y., HongZhang M. J., Zhang Y. Q. (2020). The nutritional status of pediatric patients with single ventricle undergoing a bidirectional glenn procedure. *Pediatric Cardiology*.

